The article "The Effect of Exercise Motivation on Eating Disorders in Bodybuilders in Social Networks: The Mediating Role of State Anxiety" was published in 2022. Journal: Comput Math Methods Med.

# The Effect of Exercise Motivation on Eating Disorders in Bodybuilders in Social Networks: The Mediating Role of State Anxiety

**DOI:** 10.1155/2022/7426601

**Published:** 2022-08-05

**Authors:** Yixin Liu, Yuping Cao

**Affiliations:** College of Physical Education, Xinjiang Normal University, Urumqi 830054, China

## Abstract

The aim of this study is to explore the relationship between exercise motivation and eating disorder and the mediating effect of anxiety in physical exercise. Athletes are in a social network, and the different human-machine relationships and situations generated in this may produce different sports motivations and anxiety states for athletes. The exercise motivation, status-trait anxiety, and eating disorder of 1076 fitness subjects were described and analyzed by questionnaire survey, and the survey data were statistically analyzed by means of correlation, regression, and structural equation model. The results showed that the overall detection rate of eating disorder was 56.3%. The overall detection rate of eating disorder was different between males and females. Exercise motivation has a significant positive correlation with state anxiety and eating disorder. Exercise motivation has a significant positive predictive effect on eating disorder, exercise motivation has a significant positive predictive effect on state anxiety, and state anxiety has a significant positive predictive effect on eating disorder. The mediating effect shows that state anxiety can partially mediate the relationship between exercise motivation and eating disorder, exercise motivation has a direct impact on eating disorder, and state anxiety has an indirect impact on eating disorder. In physical exercise, the exercisers' bad exercise motivation will produce too much anxiety. Poor exercise motivation and anxiety can lead to symptoms of eating disorders. In physical exercise, we should adopt reasonable value orientation and positive psychological suggestion and encourage healthy and reasonable eating behavior, which will help to prevent and treat eating disorders.

## 1. Introduction

According to the report of the American Psychiatric Association (APA) in 2000, eating disorders have become the third chronic disease among adolescent women, with the incidence rate of about 5%. Including China, Japan, South Korea, and other economically developed eastern countries, the incidence of eating disorders is reported to be increasing year by year [1]. Eating disorder (ED) abnormal eating behavior patterns, such as repeated overeating, or a type of mental disorder with diet as the main clinical characteristics is a kind of psychological disorder, involving persistent disorders in eating habits or other behaviors designed to control weight, body shape, or shape [2]. There are four main categories of eating disorders, including anorexia nervosa (AN), bulimia nervosa (BN), atypical nervosa, and binge eating disorder (BED), with anorexia and bulimia as the most common disorders. Eating disorders not only impaired physiological function but also highlight the psychological problems of patients. Excessive attention to weight and body shape as well as morbid fear of weight gain is the core features of eating disorders [3]. The origin of eating disorders is widely recognized as a result of multiple factors, with individual risk factors that must be considered in a complex etiological model, including biological factors related to personality traits, heredity and malnutrition, sociocultural factors based on cultural constraints, and family factors based on overprotection and family conflict, and in individuals, only a few studies have reported that eating disorders were associated with adverse life events prior to their occurrence, such as loss of a close relative or separation from a close friend. Again, this does not seem to be unique to patients with eating disorders, but it also stands out in individuals with other psychological problems. Further risk factors include chronic physical conditions such as diabetes, chronic intestinal disease, and other physical conditions associated with diet and body weight change [4]. Eating disorders often cause harmful manifestations of a series of physical and mental health problems (such as dehydration, arrhythmia, hypotension, decreased self-confidence, anxiety, depression, and even suicide). Therefore, identifying various precipitating factors and the mechanisms that induce eating disorders have become the key issues in the current study of eating disorders.

Studies have shown that participating in sports will bring health, self-esteem, self-confidence, and skill development, and social function brings many benefits [5, 6]. However, some aspects of sports competitions and training may damage the physical and mental health of athletes. The sports environment emphasizes physical development and training as well as nutritional strategies and diet to optimize performance, which may increase the risk of athletes suffering from eating disorders. In addition, the types of exercise motivation are often related to the sport field in which they work, and the need for specific body shape conditions or weight requirements in athletic achievement is related to the increased risk of eating disorders [7, 8]. Thus, there is a correlation between exercise motivation and eating disorders. Many behavioral characteristics describe that the extrinsic motivation and active individuals are related to eating disorders. Individuals with symptoms or diseases of eating disorders often show a high level of ineffectiveness, helplessness, lack of control, and lack of self-esteem [9]. According to the research report by Filaire et al. [10], eating disorders are related to motivation orientation. In gymnasts, an energy gap is usually caused to improve sports goals and performance. In addition, the intervention of extrinsic motivation has a negative relationship with self-esteem and body image. People with high level of extrinsic motivation will show low self-esteem and less satisfactory body image. In this group with higher self-demand, the risk of eating disorders will also increase when the body weight is low [11]. At the same time, according to the results of Homan et al. [12], they found that when teenagers' exercise motivation is to find strong sensory stimulation in sports, they may appear after 20 months having eating disorders; thus, extrinsic motivation and goal motivation are important factors that affect the occurrence of eating disorders in adolescents. However, Calderon et al. [13] learned from the survey of female college athletes that exercise motivation was also highly correlated with eating disorders. Athletes in high-intensity sports (such as basketball and cross-country running) and sports with high requirements for body shape or specific weight (i.e., cheerleading, track and field, and gymnastics) were more likely to have eating disorders in their motivation to participate in sports. That is to say, among the athletes who participated in the above sports, their intrinsic motivation was related to a lower risk of eating disorders, and their extrinsic motivation was related to a higher risk of eating disorders.

In addition, many studies have shown that negative emotions can also have a significant impact on eating disorders. They often confuse emotional state with hunger and satiety, thus relieving anxiety through eating. Environmental factors are one of the important factors affecting ED. For young people (teenagers) with a tendency to overeat, when they live in an obese family environment, they are more likely to relieve anxiety by eating. It has also been verified that physical dissatisfaction and anxiety during adolescence increase the risk of persistent obesity [14]. However, research results by Ackard et al. [15] provide strong and consistent evidence that the dieting frequency of young female college students with normal weight is related to more symptoms and more severe eating disorder behaviors and emotional distress regardless of BMI. The frequency of dieting was also associated with affective disorders such as depression, low self-esteem, difficulty in distinguishing and regulating emotions, mature fear, ineffectiveness, perfectionism, and insecurity. In domestic studies, Chen et al. [16] proposed in a study on negative emotions, overweight or obesity, and abnormal eating behavior that strong negative emotions, such as anxiety, may have a predictive effect on the occurrence of eating disorders. At the same time, exercise motivation also has a significant impact on anxiety. The relationship between exercise motivation and anxiety is mainly reflected in the higher level of motivation which will lead to higher exercise anxiety. Han [17] through the study of women's volleyball athlete exercise motivation understands that the root cause of anxiety lies in the uncertainty of the result of the game. If you have a strong desire to win and do not know what your performance will be in the upcoming competition and whether you can cope with possible difficulties in the competition, you may have high anxiety. Factors such as one's own ability, the evaluation of the importance of the competition, and the level of preparation for the competition may be related to the anxiety experience before the competition. In the research of Ye [18], the exercise motivation of amateur athletes was highly correlated with trait anxiety, and the participation motivation of sports activities significantly predicted the trait anxiety of participants. Amateur sports for sports learned helplessness is a threat to self-esteem anxiety situation.

In summary, according to previous studies, exercise motivation and anxiety can lead to eating disorders, but its internal mechanism is still unclear. At present, there is no conclusion on the relationship between the exercise motivation and eating disorders. In this study, we introduced anxiety into the effect of exercise motivation on eating disorders, aiming to determine how exercise motivation causes eating disorders. In the study, exercisers completed three tests: exercise motivation, eating disorder, and state-trait Anxiety. We assume that exercisers have a high level of exercise motivation, and exercise motivation can also lead to eating disorders, but the introduction of anxiety will reduce the impact of exercise motivation on eating disorders; that is, anxiety plays an intermediary role in the impact of exercise motivation on eating disorders. The determination of the above relationship can clarify how exercise motivation causes eating disorders on the one hand and strengthen the intervention and regulation of exercisers' anxiety on the other hand, which is of important practical significance for the prevention and treatment of eating disorders.

## 2. Objects and Methods

### 2.1. Objects

Using a convenient sampling method, 606 subjects with eating disorders were selected from 1076 subjects in 5 gymnasiums in Urumqi, including 365 males and 242 females, with the average age of 25.7 ± 3.07 years old and the average number of exercises per week of 5.65 ± 0.65. A questionnaire survey was conducted on May 4, 2020. The questionnaire collection followed the voluntary principle, and a total of 1076 questionnaires were collected. No questionnaire was collected, so no tracking was required.

### 2.2. Questionnaire Survey Method

#### 2.2.1. State Anxiety Scale

S-AI [19] is a subscale of the State-Trait Anxiety Scale (STAI) developed by Spielberger in 1983 and is one of the most widely used scales for studying anxiety and other issues in China and abroad. The questionnaire consisted of 20 items with a 4-point scoring method. Cronbach's reliability coefficient and test-retest reliability of the scale were 0.88 and 0.864, respectively. The results of confirmatory factor analysis showed that *x*^2^/df = 9.77, RMSEA = 0.07, GFI = 0.91, NFI = 0.93, CFI = 0.93, and IFI = 0.91, indicating a good structural validity. It has good reliability and validity.

#### 2.2.2. Exercise Motivation Scale

The exercise motivation scale (MPAM-R) [20] adopted the simplified version of the exercise motivation scale revised by Chen in 2013, which was reduced to 15 topics, including five dimensions of fun, ability, appearance, health, and social interaction. The scale was scored using the Likert 5-level scale, and the motivation intensity ranged from “none” to “very strong.” Cronbach's reliability coefficient of the five subscales is above 0.7, and the test-retest reliability is 0.91. The results of confirmatory factor analysis showed that *x*^2^/df = 7.63, RMSEA = 0.06, GFI = 0.92, NFI = 0.92, CFI = 0.98, and IFI = 0.93. The results of confirmatory factor analysis showed that the scale had good structural validity, indicating that the scale had good reliability and validity [20].

#### 2.2.3. Eating Disorder Scale

The Eating Disorder Attitude Test (EAT-26) [21] consisted of 26 questions with three dimensions: diet, oral control, and gluttony, which was rated on the Richter 6-point scale, ranging from 1 (always) to 6 (never). Eating disorders with a score greater than or equal to 20 were considered “at risk.” It is useful and effective in determining the prevalence of eating disorders but does not diagnose specific disorders. The index of Cronbach in this study was *α* coefficient of 0.91. The results of confirmatory factor analysis showed that *x*^2^/df = 8.92, RMSEA = 0.08, GFI = 0.94, NFI = 0.91, CFI = 0.94, and IFI = 0.92, showing good structural validity. EAT-26 has been verified as a reliable and effective tool for screening for eating disorders [22, 23].

### 2.3. Mathematical Statistics

The SPSS24.0 and AMOS24.0 analysis software packages were used for data management and statistical analysis. The demographic variables of exercisers, exercise motivation, state anxiety, and eating disorders were described in statistical analysis, difference test, correlation analysis, and regression analysis, and the structural equation model was used to test the relationship between exercise motivation, state anxiety, and eating disorders.

## 3. Results

### 3.1. Common Method Deviation Inspection

In this study, all the data were collected through a questionnaire using an anonymous questionnaire, balanced project sequence, and different measurement methods.

The test and other program control method [24], so the common method deviation (Harman single factor test) was used to test. The results show that there are seven factors whose eigenvalues are greater than 1, and the variance explained by the first factor is 18.32%, which is less than the critical criterion of 40%, indicating that there is no serious problem of common method deviation.

### 3.2. Narrative Statistical Results

Table 1 presents the mean (*M*), standard deviation (SD), and correlation matrices for exercise motivation, state anxiety, and eating disorders. The results showed that exercisers with dysphagia (25.48 ± 1.890) had higher state anxiety (71.53 ± 22.706) and stronger exercise motivation (60.89 ± 9.897) at the same time. Correlation analysis showed a significant positive correlation between state anxiety and eating disorders (*r* = 0.503, *P* < 0.01). There was a significant positive correlation between eating disorders and exercise motivation (*r* = 0.137, *P* < 0.01). There was a positive correlation between exercise motivation and state anxiety (*r* = 0.084, *P* < 0.05). In addition, there were significant differences in state anxiety (*t* = 0.460, *P* < 0.05) and eating disorders (*t* = −5.229, *P* < 0.01) between the sexes, but there was no significant difference in exercise motivation (*t* = −0.498, *P* > 0.05), so gender was not taken as the control variable in the later analysis. The above results indicated that regression analysis could be further conducted.

### 3.3. Regression Analysis of State Anxiety, Exercise Motivation, and Eating Disorder

The intermediary effect test procedure proposed by Wen et al. [25] was used to test the relationship between eating disorder (EAT) as a dependent variable, exercise motivation (MPAM-R) as an independent variable, and state anxiety (S-AI) as an intermediary variable. In the first step, the independent variable MPAM-R is tested for predicting the dependent variable EAT. The results showed that MPAM-R could explain 1.7% variation of EAT, and exercise motivation of exercisers could significantly positively predict eating disorders (*β* = 0.313, *P* < 0.01). In the second step, the prediction effect of independent variable MPAM-R on intermediate variable S-AI is examined. The results showed that MPAM-R could explain 0.5% variation of S-AI, and exercise motivation of exercisers could significantly positively predict state anxiety (*β* = 0.069, *P* < 0.05). In the third step, the prediction effects of independent variable MPAM-R and intermediate variable S-AI on dependent variable EAT are tested simultaneously. The results showed that MPAM-R and S-AI could explain 2.6% variation of EAT, exercisers' intermediary variable S-AI could significantly positively predict eating disorder (*β* = 1.366, *P* < 0.01), and the standard regression coefficient of exercise motivation on eating disorder changed from 0.313 to 1.366, but it was still at a significant level as shown in Table 2.

### 3.4. Path Analysis

First, according to the research assumptions and regression analysis, the relationship model of exercise motivation, state anxiety, and eating disorders was constructed. Exercise motivation could significantly positively predict eating disorders, exercise motivation significantly positively predicted state anxiety, and state anxiety significantly positively predicted eating disorders. Then, AMOS24.0 was used to fit the data. The fitting results are shown in Table 3 and Figure 1. In this study, CMIN/DF was 1.919, GFI, TLI, CFI, and IFI were all greater than 0.9, and RMSEA was less than 0.5. The fitting indexes all met the criteria. The above fitting indexes indicated that the model constructed in this study was good, and the relationship between exercise motivation, state anxiety, and eating disorder could be explained based on the model in Table 3 and Figure 1.

From the results of path analysis, exercise motivation had a significant and direct positive prediction effect on state anxiety (*β* = 0.05, *P* < 0.05). State anxiety had a significant direct positive prediction of eating disorders (*β* = 0.05, *P* < 0.05). Exercise motivation had a significant positive prediction of eating disorders (*β* = 0.07, *P* < 0.05). The state anxiety in this model played a part of the intermediary role.

## 4. Discussion

### 4.1. The Relationship between Exercise Motivation and Eating Disorders

This study showed that in the regular exercise population, the exercise motivation of exercisers had a significant positive prediction of eating disorders, which was consistent with the hypothesis of this study. The causes of eating disorders are very complex. Studies have shown that neurobiological factors, sociological factors, family factors, and individual psychological factors are all factors contributing to eating disorders. Bad exercise motivation, as a psychological factor, is also an important factor inducing eating disorders. This result is similar to that of Maugendre et al. [11], in that the purpose and mobility of sports affect the severity of eating disorders in exercisers who participate in intensive sports. Exercisers want to achieve the high level stipulated in the sports, which prompted them to put forward very high requirements for themselves, in order to achieve a high level of state and to strengthen the physical fitness. This kind of external motivation intervention makes the psychological and physical image have a negative relationship; with a high level of external motivation, people will show low self-esteem and less satisfactory physical image, which leads to an increase in the risk of eating disorders, but individuals do not think that this behavior is negative. In general, people who exercised regularly had higher characteristics of health motivation, ability motivation, appearance motivation, social motivation, and fun motivation. The effects of different motivation types on eating disorders were different, and the severity of eating disorders was determined with the duration of time.

### 4.2. The Relationship between Exercise Motivation and State Anxiety

This study showed that in the regular exercise population, the exercise motivation of exercisers had a significant positive predictive effect on state anxiety, which was consistent with the hypothesis of this study. Exercise motivation that is too weak or too strong will not smoothly complete the task and achieve ideal results; the former will reduce the level of individual emotional excitement and be easy to cause concentration to be easily interfered by irrelevant stimuli. On the contrary, the latter excessively focuses consciousness on specific goals and produces anxiety, which will affect individual motor performance. Understand that anxiety may originate from focusing on whether or not a goal is being achieved. If you have a strong purpose and are not sure whether you can deal with the difficulties that may occur in the exercise and whether the effect is significant after the exercise, anxiety may occur. Similar to amateur athletes, exercise motivation is highly correlated with anxiety, especially for learned helplessness athletes who take part in sports; sports is an anxiety situation threatening their self-esteem [18]. Similarly, among exercisers, women with physical anxiety will not participate in physical exercise due to negative evaluation of others, especially among young women; anxiety has become an obstacle to participate in exercise [26]. In addition, some survey results show that people with high BMI and social anxiety are more likely to avoid sports [27], so the relationship between sports motivation and anxiety needs further study.

### 4.3. The Intermediary Role of State Anxiety

The results of this study showed that among exercisers, state anxiety played a part of the intermediary role in the relationship between exercise motivation and eating disorders. Exercise motivation not only has a direct effect on eating disorders but also has an indirect effect on eating disorders through state anxiety. The results of this study explained that exercisers with higher exercise motivation were often accompanied by anxiety, and at the same time, this group of people had higher appearance, ability, social interaction, fun, and health motivation. These motivations lead to anxiety and demanding eating behaviors. At the same time, this excessive psychological pressure will have an impact on body shape, extreme eating behaviors (anorexia, bulimia, etc.), and exercise behavior itself, resulting in individuals showing a high level of ineffectiveness, helplessness, lack of control, and lack of self-esteem, indicating that negative emotions have a significant impact on eating disorders. They usually connect the emotional state with hunger and satiety, so as to relieve anxiety through eating.

## 5. Conclusions and Recommendations

### 5.1. Conclusion

(1) The total detection rate of eating disorders among exercisers is 56.3%, which is more than half, indicating that the prevalence of eating disorders is higher in the population with regular exercise. (2) Gender has significant difference in eating disorders, and the prevalence of male is higher in women, which is different from the previous research results, indicating that the male population cannot be ignored. (3) Correlation analysis shows that there is a significant positive correlation among exercise motivation, state anxiety, and eating disorder, indicating that exercise motivation of exercisers is often closely related to state anxiety and eating disorder. (4) The intermediary effect results show that state anxiety plays a partial intermediary role between exercise motivation and eating disorders. Exercise motivation indirectly affects eating disorders through state anxiety

### 5.2. Recommendations

The results of this study indicated that exercisers were among the high risk population of eating disorders, which resulted in this result because of wrong views on exercise and diet. For exercisers with eating disorders, scientific views on exercise, diet, and psychological counseling were urgently needed from professionals. At present, as a result of the popular aesthetic standards in the society, women regard thinness as their beauty and men pursue the acme figure. This requires the family, school, and society to establish a healthy and reasonable value orientation for teenagers, instead of an extreme and unique aesthetic standard. This article provides a preliminary survey of state anxiety, eating disorders, and exercise motivation that, if left untreated, eating may still plague those who want to be happy but miserable. However, the harmfulness of eating disorder goes beyond this. Psychological education on motor dysfunction should be provided for this group of people, and they should be aware that this is not as important as imagined to reduce negative emotions. Future studies should continue to investigate the relationship between the components of dysfunctional locomotion and eating disorders and explore the effects of different forms of exercise on exercise motivation, eating disorders, and anxiety. In addition, studies should include a more diverse sample size to ensure replicable studies. Also, the analysis of typical individual cases should be carried out. It is hoped that future studies will continue to investigate the influencing factors of exercise and diet in order to create more targeted treatments.

## Figures and Tables

**Figure 1:** Relationship model of exercise addiction, state anxiety, and eating disorder.

**Table 1:** Average score of all variables, the standard deviation, and the correlation coefficient.

Variable	*M* ± SD	S-AI	EAT	MPAM-R
S-AI	46.77 ± 8.165	1	0.503^∗∗^	0.084^∗^
EAT	71.46 ± 22.527	0.503^∗∗^	1	0.137^∗∗^
MPAM-R	60.96 ± 9.879	0.084^∗^	0.137^∗∗^	1

Note: S-AI: state anxiety; EAT: eating disorders; MPAM-R: training motivation. *N* = 606. ^∗^*P* < 0.05, ^∗∗^*P* < 0.01: the same below.

**Table 2:** Regression analysis of the influence of exercise motivation and state anxiety on eating disorder.

	The first step		The second step		The third step	
	Eating disorders		State anxiety		Eating disorders	
Fitting index	*β*	*t*	*β*	*t*	*β*	*t*
Training motivation	0.313	3.405^∗∗^				
Training motivation			*β* = 0.069	2.067^∗^		
Exercise motivation and state anxiety					*β* = 0.218	2.727^∗∗^
					*β* = 1.366	14.110^∗∗^
*F*	11.592		4.274		17.249	
*R*	0.137		0.084		0.512	
*R* ^2^	0.017		0.005		0.260	

**Table 3:** Model fitting index.

Model	CMIN	DF	CMIN/DF	GFI	CFI	IFI	RMSEA
Model	47.967	25	1.919	0.981	0.991	0.991	0.039

Note: ellipse represents latent variable, and box represents observed variable. The arrow between the ellipse and the box indicates the factor load, and the arrow between the ellipses indicates the path coefficient.

## Data Availability

The datasets used and analyzed during the current study are available from the corresponding author on reasonable request.
